The article "An Intelligent Clinical Psychological Assessment Method Based on AHP-LSSVR Model" was published in 2022. Journal: Comput Intell Neurosci.

# An Intelligent Clinical Psychological Assessment Method Based on AHP-LSSVR Model

**DOI:** 10.1155/2022/7584675

**Published:** 2022-03-30

**Authors:** Junli Su, Dongyang Wang

**Affiliations:** ^1^Department of Elementary Education, Jiaozuo Teachers College, Jiaozuo, Henan 454002, China; ^2^Center for International Education, Philippine Christian University, Manila 1006, Philippines; ^3^Department of Foreign Languages, Shangqiu Normal University, Shangqiu, Henan 476000, China

## Abstract

Clinical psychology is a branch of applied psychology. Clinical psychology has a clear understanding of individual behavior ability and behavior characteristics through psychological measurement analysis, observation, and other methods and combines the situation learned from individual psychosomatic diagnosis and life history with the observation and analysis of individual living conditions. Psychological quality and its evaluation methods have been widely used in many fields, which has greatly promoted the development of this field. However, the current assessment methods are mainly based on a simple statistical analysis, and the results are not accurate. To this end, this article proposes the analytic hierarchy process (AHP) and least-squares support vector regression algorithm (LSSVR). Specifically, through the construction of the specific object's psychological quality evaluation index system, the design and implementation of the psychological quality evaluation model based on AHP-LSSVR and the proposed method were discussed in the experiment.

## 1. Introduction

With the development of economy and society, people's basic life is satisfied, and they begin to put forward higher requirements and standards for health. People pay attention to physical health and pay more and more attention to mental health. Mental health has become one of the key indicators to measure people's health levels [1]. At present, most mental health assessment in China is completed by existing mental health assessment tools. Many psychological experts analyze and study people's mental health status through existing mental health assessment tools. Mental health assessment tools will be updated and improved according to the mental health of people in different periods so that the assessment results are more accurate [2–5].

With the rapid development of the Internet today, big data, cloud computing, and other information technologies have been integrated into all aspects of people's lives. People produce a large amount of data every day, and data have become a basic resource from a simple processing object [6]. Under the influence of visual analysis, many characteristics of mental health begin to appear, but the research on this aspect is still in its infancy [7, 8].

The article "An Intelligent Clinical Psychological Assessment Method Based on AHP-LSSVR Model" was published in 2022. Journal: Comput Intell Neurosci.

The research and assistance in clinical psychology are focused on individuals who are mentally ill, adjusted, or disabled, that is, individuals who have psychological problems that cause distress in their social life and their own lives. Misfortune or feeling an uncomfortable feeling and confusion or difficulty in actions, not words, and in life and even serious psychological barriers of clinical psychology are the two important areas of diagnosis and therapy. The ultimate goal is to have not adapted to people with mental distress on aid and help them to restore psychological or mental health status. The psychological adaptation and personality development of the assisted are the fundamental goals. Clinical psychology has been established so far, its development field and research topic theory and method and research and application of many aspects have been extremely large expansion, it and other branches of psychology cross and fusion are also increasing, and a lot of new topics are constantly appearing [9–11].

The theory and practice of contemporary clinical psychology are mainly composed of three frameworks: psychodynamic theory, learning theory, and humanistic theory. These three theoretical frameworks have different research orientations: psychoanalysis theory provides many dynamic approaches for clinical practice and research. Learning theory provides the basis for a large number of behavioral pathways. Humanist theory suggests some experimental approaches. The theoretical model has important practical value in clinical psychology; it can help clinical psychologist effectively organize their understanding and analysis of the behavior, to guide their decisions to make a clinical intervention; with being familiar to members of the system to communicate their results, you can also put a lot of seemingly unrelated information and data [12, 13]. Clinical psychology of dynamics theory of the basic point is that human behavior is determined by the psychological interaction of power; in this theory, the balance is in constant conflict of human needs, reality, and individual personality characteristics and responses; the individual cannot seek this balance or failure will directly lead to anxiety to seek a balance. The behavioral theory of clinical psychology is based on the assumption that all behaviors, whether normal or abnormal, are learned and that any model of psychotherapy addresses the patient's maladjustment of coping experience and the maladjustment resulting from bad habits [14]. The phenomenological model of recognizing individual uniqueness produced by experience with righteousness does not focus on individual personality structure and living habits; attention is focused on the study of individual qualities and positive publicity of the individual and individual living environment to the above [15–18].

The article "An Intelligent Clinical Psychological Assessment Method Based on AHP-LSSVR Model" was published in 2022. Journal: Comput Intell Neurosci.

## 2. Related Work

For mental health standards of this complex problem, psychology workers have done a lot of research. Still, so far, there is no ideal to known standards of domestic and international numerous psychologists, and the angle of observation and understanding of the meaning of the mental health level is different; they have put forward the psychological health standard of structure and dimension. From the comparative analysis, it can be found that they are proposed from different perspectives. Foley et al. [19] believed that it was obviously inappropriate to apply the usual mental health standards to prisoners in prison and proposed that the evaluation criteria for prisoners' mental health included the sense of security. Have a proper understanding of yourself and make a correct evaluation of the source of your crime. Based on the analysis and research of the components of civil servants' psychological quality, Wright et al. [20] put forward that the core idea of psychological quality assessment in civil servants' interview process is the standardization of psychological quality assessment, direct assessment of the internal structure of psychological quality, and indirect assessment of external indicators. Chandler et al. [21] used visual analysis technology to study the eye movement data of autistic children. They output the tracked eye movement data to MATLAB and then analyze it, trying to understand how autistic children interact with the outside world. As shown in Figure 1, the tracking 3D eye movement data are presented in the 2D visualized graph.

Some scholars have applied visualization technology to psychological assessment, breaking the traditional psychological assessment methods and opening up a new field of remote psychological analysis and assessment using the Internet [22]. However, the existing remote video system of mental health education still has problems, such as dealing with the crisis of teacher-student interaction. In order to solve the above problems, scholars have carried out research and exploration on the multichannel remote visualization of mental health education. The application of visualization technology in physical and mental health detection and evaluation is another important research topic of visualization in physical and mental health education, and its research results are very lacking [23–25]. At present, scholars only apply visualization technology to the presentation of data results. Zimmermann et al. [26] found in their research on the mental health of famous prisoners that the detection rate of mentally unhealthy prisoners in this special group was much higher than the detection rate of the general group measured by the same test and also higher than the detection rate of some other high-risk groups of mental health. Haynes ‘s [27] study found that the degree of psychological stress response of prisoners was related to the negative automatic thinking coping style, social support, and personality characteristics, as well as the degree of education, family economic illness, and the length of time served in prison.

The article "An Intelligent Clinical Psychological Assessment Method Based on AHP-LSSVR Model" was published in 2022. Journal: Comput Intell Neurosci.

From the above analysis, cognitive visualization is to use the characteristics of visualization to study the recessive characteristics. Since visualization technology has been applied to psychological assessment, it has made a breakthrough in this field. Yaxley et al. [28] used visual analysis technology to study the human cognitive framework. The study constructs a top-down framework of cognitive processes in reasoning and understanding and identifies six key points that influence human cognition. Cooney et al. [29] analyzed and studied the comprehensive evaluation method of the psychological quality detection index of motor vehicle drivers, constructed the detection index system through the expert consultation method, established the comprehensive evaluation equation of driver psychological measurement index based on analytic hierarchy process, and verified its correctness and effectiveness. Based on the analysis and research of the constitutive elements of civil servants' psychological quality, Laverdière et al. [30] proposed that the core idea of psychological quality assessment in civil servants' interview process is the direct assessment of the standardized internal structure of psychological quality and indirect assessment of externalized indicators. Williamson et al. [31] used the methods of personality test drawing person test and handwriting analysis to set up a discriminant model of the special psychological quality of sales staff in pharmaceutical factories and then evaluated and analyzed it. The above method is based on the psychological quality structure of a specific group to establish a special psychological quality discrimination model, which has strong pertinence and is not suitable for large-scale users [32, 33].

The contributions of this article are concluded as follows: (1) through the above analysis, scholars gradually realize the importance of psychological quality research; (2) some achievements have been made in the research, and the systematic psychological diathesis theory is becoming mature; (3) however, there are few researches on the psychological quality of special groups by combined methods. Therefore, the research of this article is still a blank, which has great theoretical research and practical application value [34].

The article "An Intelligent Clinical Psychological Assessment Method Based on AHP-LSSVR Model" was published in 2022. Journal: Comput Intell Neurosci.

This article consists of five parts. The first and second parts give the research status and background. The third part is the clinical psychological assessment method based on the LSSVR model. The fourth part shows the experimental results. The experimental results of this article are introduced, compared, and analyzed with relevant comparison algorithms. Finally, the fifth part concludes the full article.

## 3. Clinical Psychological Assessment Method Based on LSSVR Model

### 3.1. Clinical Psychological Assessment Process

This section proposes an evaluation model based on the analytic hierarchy process and the least-square support vector regression method to evaluate clinical psychological quality [35]. Firstly, combined with the psychological quality of the subjects, the hierarchy analysis evaluation model (AHP) was established based on the characteristic dimension judgment matrix. Secondly, this section uses a questionnaire to construct learning samples and builds a prediction model based on the LSSVR algorithm. Finally, the AHP-LSSVR psychological assessment model based on the combination of AHP and LSSVR algorithm is obtained, as shown in Figure 2.

The figure is composed of model training and model prediction and evaluation:

1. Expert evaluation module: one is to invite 15 expert group members to analyze and study 12 evaluation indicators and 1000 questions, give the relative importance ratio of the two factors before and after the AHP model according to the 1–9 scale method, and construct judgment matrix. Second, score and mark the samples required by the LSSVR model.
2. Constructing multilevel judgment matrix module: this module is to matrix the ratio of the importance of factors given by experts and calculate the maximum feature root and feature vector.
3. Consistency test module: perform mathematical calculation on the five constructed judgment matrices to verify consistency. If the verification fails, the results will be fed back to the expert group in time to revise the value of the judgment matrix until the uniformity test is met.
4. Solving the least-squares support vector machine matrix: solving the model by collecting and sorting 1000 samples of psychological quality data.
5. Constructing the LSSVR model module: construct prediction model through support vector.

### 3.2. LSSVR Model

LSSVR model transforms the inequality constraint of the support vector machine into an equality constraint problem, which greatly facilitates the solution of the Lagrange multiplier [36, 37]. The original QP problem is transformed into a problem of solving linear equations. For the support vector machine model, the constraints are the following inequality constraints:

(1) $$\begin{array}{c} \min_{\omega ,b,\xi }J\left(\omega ,\xi \right)=\frac{1}{2}\omega^{T}\omega +c\sum_{k=1}^{N}\xi_{k},\\ \text{s}.\text{t}.\;y_{k}\left[\omega^{T}\varphi \left(x_{k}\right)+b\right]\geq 1-\xi_{k},\;k=1,\ldots ,N. \end{array}$$

Furthermore, the fuzzy term of inequality constraint problem is introduced into the least-square method:

(2) $$\begin{array}{c} \min_{\omega ,b,e}J\left(\omega ,e\right)=\frac{1}{2}\omega^{T}\omega +\frac{1}{2}\gamma \sum_{k=1}^{N}e_{k}^{2},\\ \text{s}.\text{t}.\;y_{k}=\omega^{T}\varphi \left(x_{k}\right)+b+e_{k},\;k=1,\ldots ,N. \end{array}$$

Then, the Lagrange multiplier method is used to obtain the following formula:

(3) $$\begin{array}{c} L\left(\omega ,b,e;\alpha \right)=J\left(\omega ,e\right)-\sum_{k=1}^{N}\alpha_{k}\left\{\omega^{T}\varphi \left(x_{k}\right)-b+e_{k}-y_{k}\right\}. \end{array}$$

The parameters in the above equation are solved and the linear equations are obtained:

(4) $$\begin{array}{c} \left[\begin{array}{cc} 0 & 1_{v}^{T}\\ 1_{v} & \frac{\Omega +I}{y} \end{array}\right]\left[\begin{array}{c} b\\ \alpha \end{array}\right]=\left[\begin{array}{c} 0\\ y \end{array}\right]. \end{array}$$

The function matrix in the formula can be expressed as follows:

(5) $$\begin{array}{c} \Omega_{kl}=\varphi {\left(x_{k}\right)}^{T}\varphi \left(x_{l}\right)=K\left(x_{k},x_{l}\right),\;k,l=1,\ldots N. \end{array}$$

To ensure that variance is positive, that is, variance exists and is finite:

(6) $$\begin{array}{c} \sum_{i=1}^{\max\left(p,q\right)}\left(\alpha_{i}+\beta_{i}\right)<1. \end{array}$$

Finally, LSSVR is expressed as follows:

(7) $$\begin{array}{c} y\left(x\right)=\sum_{k=1}^{N}\alpha_{k}K\left(x,x_{k}\right)+b. \end{array}$$

In the application of the least-squares support vector machine to regression problems, the selection of proper kernel function is the key factor. According to the characteristics of solving problems, verified kernel function should be used instead of the inner product. Kernel function operation will transform the dot product operation of the high-dimensional feature space to the low-dimensional feature original space. In practical application, the commonly used kernel functions include polynomial kernel function radial basis function (RBF) and kernel function multilayer perceptron kernel function:

(8) $$\begin{array}{c} K\left(x,x_{i}\right)={\left(x\cdot x_{i}+\theta \right)}^{d},\;d=1,2,3,\ldots ,\\ K\left(x,x_{i}\right)=\text{e}\times \left(\text{p}-\frac{{\left\|x-x_{i}\right\|}^{2}}{\gamma^{2}}\right). \end{array}$$

For the GARCH model, we also adopt the maximum likelihood method and the parameters we want to estimate, so there is condition likelihood:

(9) $$\begin{array}{c} K\left(x,x_{i}\right)=\text{ex}\left(\text{p}-\frac{{\left\|x-x_{i}\right\|}^{2}}{\gamma^{2}}\right). \end{array}$$

Since kernel parameters can reflect the complexity of the model of the least-squares support vector machine, it can be seen from the above three kernel functions that polynomial kernel function contains controllable parameters and RBF kernel function contains controllable parameters. Although the kernel function of multilayer perceptron contains controllable parameters, it has certain limitations. RBF kernel function is the correct choice when using the least-squares support vector machine to solve specific regression problems. RBF kernel function is the most widely used kernel function in support vector machines.

The article "An Intelligent Clinical Psychological Assessment Method Based on AHP-LSSVR Model" was published in 2022. Journal: Comput Intell Neurosci.

## 4. Experimental Results and Analysis

### 4.1. Introduction to Experimental Environment and Dataset

The personal data of the subjects were collected by paper questionnaire survey, which was compiled in strict accordance with the standards, requirements, and procedures of the psychological scale. The combined method of quantitative research and qualitative research was adopted. Taking 12 psychological quality evaluation index system of students established by 15 experts as the topic item, 1000 personal psychological quality scores of students were collected by organizing students to answer the questions. The questionnaire survey lasted for three weeks. Before filling in the questionnaire, students should explain the filling method and scoring method patiently and carefully. Remind the students to read the meaning of each question carefully; then according to the question, the students think of the importance of the psychological quality of the military cadets: the range of minor importance, 0–20 points; slightly important, range 21–40 points; obviously important, 41–60 points; strongly important, 61–80 points; extreme importance, 81–100 points. The higher the score is, the more important it is. The validity and reliability of the military cadets' psychological quality questionnaire have been formed, which basically achieves the research purpose.

This article evaluates the mental health grade of cadets and puts forward reasonable evaluations for individuals according to the evaluation results so as to grasp the real mental condition of cadets and provide reliable data basis for the evaluation and education of cadets' mental quality in military academies. In this study, experts were organized to manually score the psychological quality data of 1000 students. The specific method is to divide 24 experts into six groups according to each group of 4 people and divide 1000 pieces of data into six pieces. The first four groups have 170 pieces for each group, and the last two groups have 171 pieces for each group. Four experts in each group, according to the unified standard before determining the index system and questionnaire development, give the final evaluation score to the student according to the 12 questions. Each expert needs to complete the final evaluation and scoring work of all students assigned to the group.

The article "An Intelligent Clinical Psychological Assessment Method Based on AHP-LSSVR Model" was published in 2022. Journal: Comput Intell Neurosci.

The average score of the four experts is the final psychological quality evaluation score of the student. The expert scoring result is the sample set, and the least-squares support vector regression algorithm is used to construct the LSSVR prediction model. The trainees whose final evaluation score is in the extreme and significant risk range will be identified as the unqualified personnel of psychological quality, and the psychological guidance instructors of military colleges and psychologists of health departments shall provide corresponding psychological counseling and treatment to them. Students whose final evaluation score is in the medium-risk range will be identified as psychologically qualified personnel. Psychological quality can be improved by reviewing personal psychological files for targeted education and training.

### 4.2. Experimental Results Analysis

When building a model based on LSSVR, once the form of kernel function is determined, multiple hyperparameters will be adjusted accordingly in the model. The accuracy of the model is greatly affected by the value of hyperparameters. When RBF is selected as the kernel function, the hyperparameters that need to be adjusted for the LSSVR model include regularization parameter, insensitive parameter, and RBF kernel parameter. In determining the AHP-LSSVR Cadets psychological assessment model, the precision of the model to a certain extent is affected by the three parameters. A lot of methods are used to determine the parameters, but there is no relative standard method. Integrating the experimental data, this article adopts the calendar to select the parameters using mean absolute error (MAE).

Figure 3 shows the thermal diagram of model MAE experimental results when the regularization parameter and gamma are set. It can be seen from the figure that with fixed gamma, the model's overall mean absolute error decreases as the regularization parameter value increases and then stabilizes in a certain value range, but the time efficiency also increases exponentially. In the case of a fixed regularization parameter, the value of gamma will increase or decrease continuously, and the mean absolute error will decrease.

The article "An Intelligent Clinical Psychological Assessment Method Based on AHP-LSSVR Model" was published in 2022. Journal: Comput Intell Neurosci.

In psychological evaluation, it is very important to match different colors for different psychology, which is closely related to the information expression ability and aesthetics of visual results. The content of this article is based on psychology and visualization, and the choice of color is very important for these two disciplines. A reasonable color scheme can enhance users' understanding of data and deepen their interest in data exploration. In the process of development, the system in this article takes blue as the theme color, and the color in the visual view is composed of different hues, saturation, and brightness. It can conveniently select the color that one prefers or is currently suitable. According to the self-evaluation of psychological factors, the psychological conditions reflected by the 12 factors of the scale are combined with different color spaces to differentiate each factor by coloring so as to obtain various visual views, such as the scatter plot and broken line plot.  Figure 4 shows the color matching of the bundled bar chart that analyzes the data of the self-evaluation scale of psychological autism. Before and after the contrast effect can be seen, the color matching method can better display different psychological states.

The latest data analysis module helps users timely understand their current mental health status, find their own mental health problems, and make adjustments through visual analysis of the data just entered by users. The current data analysis module is not much different from the current data analysis module of the mental health assessment system established at the end of chapter 3. Only the improvement suggestions in the module are revised. When proposing improvement suggestions for users, they are not only based on the current evaluation results but also combined with the historical data analysis results of users. Historical data analysis module uses a feature selection algorithm to analyze the history of the user data for the history of this text system data analysis module and in the third chapter to establish an evaluation system of psychological health of the historical data analysis module of the larger correction. To leave the visualization scheme for total score and each factor analysis, the radar diagram and the word cloud are replaced with the scatter tree diagram to carry out the joint analysis of factors and problems.

The revised module still uses the area diagram to present the trend of the total score and uses the broken line diagram to analyze the trend of each factor. Users can view the change of factors or total scores on a specific day or period of time through the timeline.  Figure 5 shows the change of Carrie's total scores and all factors over time from April 9 to July 9. As you can see from Figure 5, Carrie's OCD score was significantly higher than the others, with the total score reaching its peak on May 26 due to a sudden increase in anxiety and depression scores. When the mouse cursor slides over the factor rectangular label in the factor line graph, the curve diagram of the corresponding factor changing with time will be drawn in the factor line graph. When the mouse cursor moves away from the factor rectangular label, the factor curve just drawn will be deleted. Click the mouse to draw the factor curve in the graph. In order to make the difference between factors clearer, you can click to select multiple factors for analysis at the same time.

The article "An Intelligent Clinical Psychological Assessment Method Based on AHP-LSSVR Model" was published in 2022. Journal: Comput Intell Neurosci.

The historical data analysis module is modified to use scatter tree graph and to use factor and visualization of the feature selection algorithm, in which the horizontal axis shows time, at a point on the timeline for each problem with the change of time, the problems and factors of ownership using wires, and the color of the points for distinguishing factor categories, and each problem belongs to the factor and the size of the point score is used to represent each problem.

Figure 6 shows the MAE experimental results of the model with different values. It can be seen from the figure that MAE error will increase gradually in the process of gradually increasing insensitive parameters. However, the gradual decrease of insensitive parameters will not bring infinite reduction of MAE, but the decrease will lead to the calculation efficiency of the model. The convergence rate decreases, so choosing an appropriate insensitive parameter value is particularly important for the efficiency and accuracy of the experiment. In this article, the insensitive parameter value is 0.0001 during the experiment.

As shown in Figure 7, we can also see that the most important factors to pay attention to are as follows: obsessive compulsive disorder, depression, and anxiety. Most of the problems in obsessive compulsive disorder factor are always in high scores, while the problems in anxiety factor fluctuate greatly, which may be caused by excessive pressure in a certain period of time or large mood fluctuations in a certain period of time. In the depression factor, both the high score and the big fluctuation exist, and the reason that the depression factor score exceeds the normal value is related to the fluctuation of the depression factor because the emergence of these fluctuations also helps to find the potential depression problems. These identified problems need to be adjusted or seek help from the nearest mental health counseling center in order to restore mental health status within the normal range.

The article "An Intelligent Clinical Psychological Assessment Method Based on AHP-LSSVR Model" was published in 2022. Journal: Comput Intell Neurosci.

In Figure 8, *∗* shows the premeasured classes of the physiologic states of university students, ○ represents the actual category of the psychological state of college students, through contrast display can directly display the psychological state of college students' cognitive results and real university students' psychological state category, wherein 1, 2, 3, 4, and 5 points show psychological health, compulsive anxiety, interpersonal relationship, and depression when *∗* and ○ overlap, the predicted category of college students' psychological state is consistent with the actual category, indicating correct recognition. When *∗* and ○ do not coincide, the predicted category of college students' psychological state is inconsistent with the actual category, and the effectiveness of the proposed method is proved.

As shown in Figure 9, the first dimension is mainly related to negative psychological emotions related to diseases, such as depression and irritability, so it is named negative emotions. The second dimension is mainly related to the impairment of interpersonal communication and daily life functions, which is named behavioral response. The content of the third dimension mainly reflects the patients' feelings and thoughts about the disease itself, so the contents of the three dimensions named as the role of the disease are consistent. For the above three newly generated dimensions, we further test their unidimensional and internal consistency system number. According to the above results, we can see that the three newly generated dimensions are barely considered to be unidimensional, and their internal consistency coefficients are also at an acceptable level.

## 5. Conclusions

This article explores the use of converged machine learning algorithms to analyze mental health data in order to understand people's mental health status and propose different feedback and suggestions based on users' mental health data. Visual analysis can help users understand their own mental health status and find any serious or potential mental health problems. In this article, the clinical psychological assessment methods based on LSSVR are analyzed, and the conceptual principles and steps of the analytic hierarchy process and least-square support vector regression algorithm are analyzed. The model evaluation method of AHP and least-square support vector regression algorithm was studied, and the psychological evaluation method of military cadets based on LSSVR was proposed. Using a wide variety of psychological assessment methods to establish the corresponding model was studied, while the psychological level assessment of a single object, but by the time relationship, students psychological quality index system research sample, is relatively small, realize the students' psychological computer data acquisition and students psychological quality evaluation system on the development and application of work have not had time to begin. However, the current psychological assessment methods are mainly aimed at a certain characteristic of the crowd. Hence, more general clinical psychological assessment methods for all populations need further study.

The article "An Intelligent Clinical Psychological Assessment Method Based on AHP-LSSVR Model" was published in 2022. Journal: Comput Intell Neurosci.

## Figures and Tables

**Figure 1:** The 2D visualized graph.

**Figure 2:** Clinical psychological assessment model based on LSSVR model.

**Figure 3:** Thermal diagram of MAE with different parameter values.

**Figure 4:** Binding bar diagram effect before and after color matching. (a) Before match colors and (b) after match colors.

**Figure 5:** Change trend of the psychological score during 2017.04.09–2017.07.09.

**Figure 6:** MAE experimental results with different values.

**Figure 7:** Results of feature selection algorithms for historical psychological data.

**Figure 8:** Results of mental state recognition based on LSSVR.

**Figure 9:** Different dimensions of negative emotion test results.

## Data Availability

The data used to support the findings of this study are available from the corresponding author upon request.
